# PerAnSel:  A  Novel Deep Neural Network-Based System for Persian Question Answering

**DOI:** 10.1155/2022/3661286

**Published:** 2022-07-18

**Authors:** Jamshid Mozafari, Arefeh Kazemi, Parham Moradi, Mohammad Ali Nematbakhsh

**Affiliations:** ^1^Big Data Research Group, Faculty of Computer Engineering, University of Isfahan, Isfahan, Iran; ^2^Department of Linguistics, Faculty of Foreign Languages, University of Isfahan, Isfahan, Iran; ^3^Department of Computer Engineering, University of Kurdistan, Sanandaj, Iran

## Abstract

Question answering (QA) systems have attracted considerable attention in recent years. They receive the user's questions in natural language and respond to them with precise answers. Most of the works on QA were initially proposed for the English language, but some research studies have recently been performed on non-English languages. Answer selection (AS) is a critical component in QA systems. To the best of our knowledge, there is no research on AS for the Persian language. Persian is a (1) free word order, (2) right-to-left, (3) morphologically rich, and (4) low-resource language. Deep learning (DL) techniques have shown promising accuracy in AS. Although DL performs very well on QA, it requires a considerable amount of annotated data for training. Many annotated datasets have been built for the AS task; most of them are exclusively in English. In order to address the need for a high-quality AS dataset in the Persian language, we present PASD; the first large-scale native AS dataset for the Persian language. To show the quality of PASD, we employed it to train state-of-the-art QA systems. We also present PerAnSel: a novel deep neural network-based system for Persian question answering. Since the Persian language is a free word-order language, in PerAnSel, we parallelize a sequential method and a transformer-based method to handle various orders in the Persian language. We then evaluate PerAnSel on three datasets: PASD, PerCQA, and WikiFA. The experimental results indicate strong performance on the Persian datasets beating state-of-the-art answer selection methods by 10.66% on PASD, 8.42% on PerCQA, and 3.08% on WikiFA datasets in terms of MRR.

## 1. Introduction

Question answering (QA) systems are a branch of artificial intelligence that employ machine learning techniques with the aim of automatically answering questions asked by humans. In general, humans investigated several ways to find answers of questions, such as asking experts and searching through text-based documents. Due to the availability of digital and nondigital text resources, it is time-consuming to investigate all of these resources to answer questions [1]. Recently, the advancement of machine learning and deep learning techniques, high computing speed, and web resources encouraged researchers to take advantage of the computer's ability to find answers among web resources [2].

Information retrieval (IR) systems were the initial types of QA systems. Traditional search engines were actually IR systems. These systems do not find the exact answer of the question; instead, they provide relevant web pages to the user, which may include answers, and the user should find the exact answers from the returned web pages. In contrast, QA systems seek to find the exact answer to the questions. Generally, QA systems can be divided into two categories: (1) knowledge-based QA systems and (2) information retrieval-based (IR-based) QA systems. Knowledge-based systems [3] deploy structured documents such as massive knowledge graphs for finding the exact answers. In these graphs, the nodes are entities—objects, events, situations, or abstract concepts—and the edges connect a pair of entities and show the relationship of interest between them. While deploying knowledge-based QA systems has shown great performance for some specific domains, building and updating knowledge graphs is a time-consuming process. IR-based QA systems [4] attempt to find the answer of a question inside unstructured documents such as web pages. These systems eliminate the need to building and updating knowledge graphs; instead, they have to deal with new challenges such as machine reading comprehension (MRC). MRC systems scan unstructured documents and extract meaning from the raw text [5].

IR-based QA systems consist of four general components: (1) question processing, (2) information retrieval, (3) answer extraction, and (4) answer selection. The question processing component extracts required information from the user's question and applies necessary modifications to the question, if needed. The information retrieval component also retrieves relevant passages to the user's question from the documents and pulls them. The answer extraction component then extracts the exact answer of the questions from the retrieved passages. The answer selection component tries to detect the best answer for the user's question. Nowadays, most of the QA systems concentrate on factoid questions, questions that can be answered with facts expressed in a few words [6].

Many QA systems have been developed for the English language [6]. Recently, some research studies have been performed for some other languages [7–9]. Most of the works on QA for non-English languages have focused on the question processing [10] and answer extraction components [11]. While it has been shown that the performance of answer selection component has a significant impact on the overall performance of a QA system [12], a limited number of research studies have been performed on the answer selection component.

To the best of our knowledge, there is no research on answer selection methods for the Persian language. About 110 million people from Iran, Tajikistan, Afghanistan, and six other countries speak Persian. Persian is a free word-order, morphologically rich, low-resource, and right-to-left language [13]. This language is written from right to left and rich in morphology. The standard word order of the Persian language is subject-object-verb (SOV), although all other orders (SVO, OSV, VSO, etc.) are acceptable. In addition to this, this language is low-resource; that is, there are not enough resources for training learning algorithms for this language. Due to being low resource of the Persian language, in this article, we generate the first large-scale native dataset for answer selection in Persian. In addition, due to being free word-order of this language, we present a novel method to address the answer selection problem in QA systems for the Persian language. In this method, we parallelize a sequential method containing convolutional neural networks (CNNs) [14] and recurrent neural networks (RNNs) [15] and transformer-based methods like bidirectional encoder representations from transformers (BERT) [16] to handle various orders in the Persian language. Moreover, to handle the morphological rich problem of the Persian language, we use the BERT language model. Özçift et al. [17] demonstrated that BERT can overcome the morphological rich problem. The following research questions were explored in this article:

- Does using a native dataset for answer selection task show better performance than using a translated dataset for the Persian language?
- Does our novel method have more appropriate performance on the native dataset than state-of-the-art methods for the Persian language?
- Is there any difference between methods for standard word order (SOV) and other word orders?
- Does multilingual BERT show better performance than monolingual BERT on the Persian language?
- Does using the output of the question processing component improve the performance of the answer selection component for the Persian language?

Since there is no large-scale native answer selection dataset for training and evaluating answer selection models for the Persian language, in this article, we generate a large-scale native dataset for the Persian language called PASD (Persian Answer Selection Dataset). The PASD contains about 20,000 questions and 100,000 question-answer pairs. In addition to this, we translate the WikiQA [18] dataset to Persian named WikiFA in order to evaluate the translation method for the Persian language.

Our method called PerAnSel is a novel method that uses two deep learning methods in parallel for the Persian language. PerAnSel consists of two components: (1) SOVWO (subject-object-verb word order) and (2) OWO (other word orders). SOVWO utilizes 1-D CNN and LSTM (long short-term memory) networks in order to handle standard word order (SOV). OWO utilizes transformer-based models in order to handle nonstandard word orders (VSO, OSV, etc.).

The contributions of this article are as follows:

- Due to the lack of a large-scale native dataset for the Persian language, we provide a large-scale native dataset for the answer selection task in the Persian language.
- We propose a novel method called PerAnSel, for answer selection in the QA systems for the Persian language. PerAnSel uses sequential models such as LSTM and 1-D CNN to process sentences with SOV word order. These algorithms are commonly used when we are dealing with sentences with SOV word order, because SOV is the standard word order of the Persian language and most of sentences are stated in this word order. PerAnSel deploys a transformer-based language model to process sentences with other word orders. The transformer-based model is composed of fully connected neural networks and attention mechanism [19], which enable it to address the morphologically problem in the Persian language [17].
- In order to address the answer selection problem for the Persian language, we use transformer-based models and sequential models in parallel.
- Inspired by Ref. [20], we present a question processing method for the Persian language. The experiments show that this improves the accuracy of QA systems.

Our dataset (PASD) and all the codes implemented in this article are freely available for public use at https://github.com/BigData-IsfahanUni/PerAnSel. First, for evaluating the performance of the proposed dataset, we implemented some state-of-the-art models and fine-tuned them with the PASD dataset. After investigating the quality of PASD, we evaluate the PerAnSel model using the PASD dataset. We achieved an MRR (mean reciprocal rank) [21] score of 92.11% using PerAnSel, which is better than state-of-the-art models.

This article is organized as follows: In Section 2, related works are described. In Section 3, the process of generating translated and native datasets are explained. In Section 4, the proposed method for the answer selection is presented. In Section 5, baseline models, implementation details, and evaluation metrics are described. In Section 6, the experiments results and discussion on answer selection and question processing methods, and error analysis are explained. Finally, the article is concluded in Section 7.

## 2. Related Works

In this section, a comprehensive survey is provided for existing answer selection studies. These studies are classified into two groups: (1) those works that build a dataset for answer selection and (2) those that proposed some answer selection methods. Here, we first present those works performed on the English language and then those methods that are proposed for the other languages.

### 2.1. English

English is a widely used languages in all over the world [22]. There are many works that have focused on the English language for QA systems.

#### 2.1.1. Datasets

One of the early datasets for the answer selection task is TrecQA. This dataset was created from the TREC-8 to TREC-13 QA tracks, which use TREC-8 to TREC-12 tracks for the training set and TREC-13 track for the dev set and test set. TrecQA consists of two different versions: the raw version and the clean version. The raw version [23], which is the first version of this dataset, contains 1229 questions for the training set, 82 questions for the dev set, and 100 questions for the test set. In the clean version [24], the questions that do not have any answers or all of the answers of the question are correct or incorrect are removed. By applying these changes, 1229 questions remain for the training set, 65 questions for the dev set, and 68 questions for the test set. To generate the training set, they used two approaches: (1) manually judgement and (2) automatic judgement. In the manually judgement approach, they employed some crowdworkers to annotate 94 questions, afterwards they named this training set TRAIN. While, in the automatic judgement approach, they leveraged automatic methods to annotate 1229 questions, and they named it TRAIN-ALL.

To create the WikiQA dataset, Yang et al. [18] employed the Bing search engine query logs. They believed that the questions searched in the search engines are more similar to real-world questions of the users. Based on this fact, they extracted some questions from the Bing query logs and detected the Wikipedia pages the questions were related to. Eventually, they generated candidates' answers from the sentences of the summary section of the related Wikipedia page. Some questions in this dataset only include incorrect candidate answers. These items are included in the original version of this dataset but are ignored in most research studies. This dataset contains 2118 questions for the training set, 296 questions for the dev set, and 633 questions for the test set.

The InsuranceQA dataset [25] is the first released dataset in the insurance field for answer selection task and collected from Insurance Library website (http://www.insurancelibrary.com). The questions are composed by real users, and the answers to the questions are high-quality answers prepared by professional users. A unique feature of this dataset is the huge number of correct candidate answers to each question. For each question, 500 candidate answers are considered. The incorrect candidate answers are the correct candidate answers to other questions. This dataset contains 12889 questions for the training set, 2000 questions for the dev set, and 2000 questions for the test set.

The SelQA dataset [26] presented a new dataset with annotated questions of various topics from Wikipedia. They eliminated the limitation of the number of questions and scopes of topics that existed in other datasets. They also proposed a new annotation scheme to create a large corpus. This dataset contains 5529 questions for the training set, 785 questions for the dev set, and 1590 questions for the test set.

#### 2.1.2. Methods

The methods proposed to solve the answer selection for the English language can be categorized into six groups: (1) feature-based, (2) Siamese-based, (3) attention-based, (4) compare-aggregate-based, (5) language model-based, and (6) other methods.

Feature-based methods utilized feature engineering on questions and candidate answers to solve the answer selection task. These methods select the final answer based on common words between the question and the candidate answers [27]. Since feature-based methods use exact match between questions' and candidate answers' words, they cannot distinguish synonymous words. Even using lexical sources such as WordNet [28] could not fix this shortcoming. Then, the dependency trees and edit distance algorithms [29, 30] were employed to feature-selection. In these methods, the candidate answers are ranked based on the increasing order of edit distance between the question dependency tree and the candidate answer dependency tree.

Siamese-based models are based on Siamese neural network architecture. Siamese neural network is a neural network that employs a shared-weight neural network to process two different input vectors to generate an output vector representation for each input [31]. In the answer selection problem, two inputs are a question sentence and a candidate answer sentence. When the output vectors are generated for the question and the candidate answer, the generated output vector representations are compared, and their relevance is calculated. Yu et al. [32] utilized the Siamese neural network and deep learning LSTM to solve the answer selection task. This model used a convolutional neural network (CNN) as the shared-weight neural network and used logistic regression to compute the relevance between the question and the candidate answer. He et al. [33] presented multi-perspective convolutional neural network (MPCNN) model. They used a CNN with multiple window sizes and multiple types of pooling as the shared-weight neural network. They also employed multiple distance functions such as cosine distance, Euclidean distance, and element-wise difference to calculate the relevance. They showed that using this model generates high-quality representation vectors for the question and the candidate answer. In this regard, Rao et al. [34] presented a novel pairwise ranking approach and implemented the MPCNN model by this approach. The authors believed that using pairwise ranking rather than using pointwise ranking leads to the generation of high-quality output vector representations for the question and the candidate answer. Kamath et al. [35] used a simple recurrent neural network (RNN) as shared-weight neural network and employed logistic regression to calculated the similarity between the question and the candidate answer. However, they showed that integrating question classification and answer selection component eliminates the requirement of a heavy-weight neural network to solve the answer selection task.

Rather than processing the question and the candidate answer separately based on the Siamese neural network architecture, attention-based models, inspired by the attention mechanism [19], use context-sensitive interaction between the question and the candidate answer to calculate the similarity. Yang et al. [36] leveraged an RNN to implement the attention mechanism for answer selection task. He et al. [37] showed that using CNNs instead of RNNs in the attention-based models leads to the generation of more high-quality output vector representation for the question and the candidate answer. Finally, Mozafari et al. [38] showed that using the attention mechanism, convolutional neural networks, and the pairwise ranking, at the same time, improves the quality of the output vector representations.

The compare-aggregate-based models follow the Compare-Aggregate framework [39]. In this framework, context-sensitive interaction between smaller units such as word units or token units is used. By aggregating the calculated values of the interactions, the relevance between the question and the candidate answer is calculated. He and Lin [40] presented the first method that uses the compare-aggregate method for answer selection. They performed word-level matching instead of sentence-level matching and used a CNN to aggregate the interaction values. Wang et al. [41] showed that word-level matching in two directions of words order of inputs, and using a BiLSTM (bidirectional LSTM) to aggregate the matching values, makes an output vector representations more meaningful than the He and Lin [40] method.

Recently, language model-based models have been widely used, and their results have shown that their performance is better than the prior methods. These models use pretrained language models instead of convolutional neural networks or recurrent neural networks. This feature enables the model to gain sufficient knowledge of source languages, and the model understands the meaning of the question and the candidate answer better. Yoon et al. [42] proposed one of the first models that use a language model to solve the answer selection task. In their research, the ELMo (embeddings from language model) language model [43] was employed. Mozafari et al. [44] showed that using recurrent neural networks on top of the language models such as BERT [16] leads to the generation of more high-quality output vectors than a mere use of language model output vector. Laskar et al. [45] showed that using heavier language models such as RobertA (robustly optimized BERT pretraining approach) [46] enhances answer selection models' performance. However, Mozafari et al. [47] showed that the weight of the language model is not a criterion to have a high-performance answer selection model. They indicated that the DistilBERT language model [48], a lighter model than the BERT language model, has a better performance. Shonibare [49] showed that various rankings, such as pairwise and triplet rankings, can improve answer selection models that utilize language models. Han et al. [50] also showed that utilizing the passages of candidate answers along with questions and candidates' answers increases the model performance.

There are some methods that are not in earlier categories. In these methods, the authors investigate novel paths to solve answer selection. Shen et al. [51] implemented the KABLSTM model. This model employed knowledge graphs; thus, they proposed a context-knowledge interactive learning architecture. Jin et al. [52] proposed a new ranking method and used a multitask learning framework.

### 2.2. Other Languages

For the Chinese language, several datasets are provided. Some of these datasets are closed domains and were created for medical purposes, whereas others are open domains. Several datasets are also provided for languages such as Portuguese and Arabic. Native and translation methods have been used for generating these datasets.

#### 2.2.1. Datasets

The cMedQA dataset [53] is a closed-domain medical dataset for the Chinese language. This dataset consists of online medical questions and answers from the XunYiWenYao website (http://www.xywy.com). This dataset contains 50,000 questions for the training set, 2,000 questions for the dev set, and 2,000 questions for the test set.

Zhang et al. [54] improved the cMedQA dataset and generated a twice number of questions. This new dataset contains 10,000 questions for the training set, 4,000 questions for the dev set, and 4,000 questions for the test set.

The cEpilepsyQA dataset [55], like the cMedQA datasets, includes XunYiWenYao website medical questions. The difference is in selecting the negative answer candidates for each question. In this dataset, negative answer candidates are more similar to the correct answer. This dataset contains 3920 questions for the training set, 490 questions for the dev set, and 490 questions for the test set.

The DBQA dataset [56] is an open-domain dataset. During producing the dataset, annotators are asked to extract a sentence from documents and generate a question for the sentence. This dataset contains 8772 questions for the training set, 5779 questions for the dev set, and 2500 questions for the test set.

The MilkQA dataset [57] is a closed-domain dataset prepared for the Portuguese language. The questions are about dairy. Some people asked the questions, each with various backgrounds, but Embrapa's customer service experts answered the questions. This dataset contains 2307 questions for the training set, 50 questions for the dev set, and 300 questions for the test set.

The WikiQAar dataset [58] is an Arabic dataset produced by translating the WikiQA dataset into Arabic. The number of questions in this dataset is the same as the WikiQA dataset.

The CQA-MD dataset [59] is a closed-domain Arabic dataset for community question answering in the domain of medical forums. This dataset is collected from WebTeb (http://www.webteb.com), Al-Tibbi (http://www.altibbi.com), and medical corner of Islamweb (http://consult.islamweb.net). This dataset contains 1031 questions for the training set, 250 questions for the dev, and 250 for the test set.

Currently, there is only a work on building native answer selection dataset for the Persian language. Jamali et al. [60] created the PerCQA (Persian Community Question Answering) dataset, a dataset for community question answering, based on questions and answers posed by users in the Ninisite (https://www.ninisite.com) forum. PerCQA contains about 692 questions for the training set, 99 questions for the dev set, and 198 questions for the test set. To the best of our knowledge, currently, there is no large-scale native QA dataset for answer selection in Persian, neither as a monolingual nor as a cross-lingual dataset. In this article, we present the first large-scale native dataset for the Persian language, called PASD. This dataset contains 17567 questions for the training set, 1000 questions for the dev set, and 1000 questions for the test set. Every question in the PASD dataset has five candidate answers.

#### 2.2.2. Methods

There are also some research studies performed on non-English languages such as Chinese and Arabic. For example, Zhang et al. [54] proposed a multiscale attentive network to capture the interaction between questions and candidate answers. Zhang et al. [61] took advantage of the Siamese neural network architecture and proposed a hybrid model by combining convolutional neural networks and recurrent neural networks. Finally, Chen et al. [55] presented the embeddings of Chinese texts in character level, and used the co-attention mechanism and fusion layer to capture the interaction between user's question and candidate answers. Almiman et al. [62] presented a weight ensemble model for Arabic language, which ensembles the output of three classification models to predict final prediction score. To the best of our knowledge, currently, there is not a method for answer selection task for the Persian language. In this article, we also present a method for answer selection for this language, called PerAnSel.

Table 1 provides a review of the datasets, and Table 2 provides a summary of the models.

## 3. Dataset

State-of-the-art models in machine learning tasks deploy deep learning algorithms. Deep learning algorithms require a considerable amount of data for training. In order to use deep learning algorithms in answer selection tasks, a large-scale dataset consisting of annotated data is required. As mentioned earlier, no research has been conducted on answer selection in the Persian language. There is also no large-scale native dataset for the answer selection task in Persian language. In this section, we describe two datasets for answer selection task in Persian language: (1) WikiFA and (2) PASD. To create the PASD dataset and implement our model, we need to use BERT language model. In the following, we describe this language model and several its derivations.

BERT [16] is a transformer-based language model published by Google. It was a revolution in the NLP (natural language processing) community in various tasks, including text classification, question answering, and natural language inference. BERT's key technical innovation is applying the bidirectional training of transformer to language modeling. Devlin et al. [16] employed the encoder of the transformer [63] to learn language representation. Transformer encoders consist of self-attention components instead of LSTMs. Unlike LSTM, the self-attention mechanism is fast to train because all the words are processed simultaneously. In transformer encoders, self-attention layers process an input simultaneously. Algorithm 1 indicates the algorithm of the BERT language model.

Assume *v* ∈ *ℝ*^*N*^ indicates an *N*-dimensional vector, and *m* ∈ *ℝ*^*N*×*M*^ indicates an *N* × *M* matrix. There are *S* self-attention layers in each encoder transformer. The *i*^th^ self-attention generates vector *Z*_*i*_ as the output. This vector is produced using three vectors—Query (*Q*_*i*_), Key (*K*_*i*_), and Value (*V*_*i*_), which are the result of the multiplication emd_*j*_, embedding vector for the *j*^th^ token, by *W*_*Q*_*i*__ ∈ *ℝ*^|emd_*j*_|×|*Q*_*i*_|^, *W*_*K*_*i*__ ∈ *ℝ*^|emd_*j*_| × |*K*_*i*_|^, and *W*_*V*_*i*__ ∈ *ℝ*^|emd_*j*_|×|*V*_*i*_|^. *W*_*Q*_*i*__, *W*_*K*_*i*__, and *W*_*V*_*i*__ are learnable parameters, which are learned during the training phase. The following equations show these operations and in (4), *σ* demonstrates the softmax function:

(1) $$\begin{array}{c} Q_{i}⇐{\text{emd}}_{j}\times W_{Q_{i}}, \end{array}$$

(2) $$\begin{array}{c} K_{i}⇐{\text{emd}}_{j}\times W_{K_{i}}, \end{array}$$

(3) $$\begin{array}{c} V_{i}⇐{\text{emd}}_{j}\times W_{V_{i}}, \end{array}$$

(4) $$\begin{array}{c} Z_{i}⇐\sigma \left(\frac{Q_{i}\times K_{i}^{T}}{\sqrt{\left|K_{i}\right|}}\right)\times V_{i}. \end{array}$$

The outputs of *Z*_1_ to *Z*_*S*_ are concatenated, and vector *Z*_1..*S*_ is produced. By multiplying *Z*_1..*S*_ by matrix *W*_*O*_ ∈ *ℝ*^*Z*_1..*S*_×768^, the final vector *Z* is produced as final output of the all self-attention layers. *W*_*O*_ is a learnable matrix. The following equation shows the multiplication:

(5) $$\begin{array}{c} Z⇐Z_{1..S}\times W_{O}. \end{array}$$

The generated vector *Z* is transferred to a multilayer perceptron, and emb_*j*_^new^ is produced. This is a new embedding vector for *j*^th^ token. *W*_*F*_ ∈ *ℝ*^|768|×|emb_*j*_|^ and *b*_*F*_ ∈ *ℝ*^|emb_*j*_|^ are learnable parameters. This multilayer perceptron is shown in the following equation:

(6) $$\begin{array}{c} {\text{emd}}_{j}^{\text{new}}⇐Z\times W_{F}+b_{F}. \end{array}$$

The emd_1..|inputs|_^new^ vectors are transferred to the next encoder. This operation is repeated to the number of encoders.

MBERT (multilingual BERT) [16] is a BERT-base language model trained on the Wikipedia documents in 104 languages using a masked language modeling (MLM) objective. The model has 177M learnable parameters. DistilmBert [48] is a distilled version of the BERT-base multilingual model. The model is trained on Wikipedia in 104 different languages. The model has 134M parameters compared to 177M parameters for MBERT. On average DistilmBERT is twice as fast as MBERT. ParsBERT [64] is a BERT-base language model, which is trained on a massive amount of public Persian corpora including Wikidumbs (https://dumps.wikimedia.org/fawiki/), MirasText (https://github.com/miras-tech/MirasText), and six other manually crawled text data with more than 3.9M documents, 73M sentences, and 1.3B words. ALBERT-Persian (A Lite BERT) [65] is an Albert base for the Persian language. The model is trained like ParsBERT on Wikidumbs, MirasText, and other crawled text data.

### 3.1. WikiFA

We build WikiFA by translating an English dataset to Persian. We create this dataset in order to evaluate the translation method for the Persian language. We use machine translation to translate the instances in WikiQA [18] to the Persian language. To this end, we deploy Google translate API and translate each record in WikiQA to Persian. Assume that each record in WikiQA is in the form *R*_*E*_={*Q*_ID, *Q*_*E*_, *D*_ID, *D*_Title, *A*_ID, *A*_*E*_, Label}, where *Q*_ID is question id, *Q*_*E*_ is English question, *D*_ID is document id, *D*_Title is document title, *A*_ID is candidate answer id, *A*_*E*_ is English candidate answer, and Label is candidate answers' label. For each record *R*_*E*_, we add *R*_*F*_={*Q*_ID, *Q*_*F*_, *D*_ID, *D*_Title, *A*_ID, *A*_*F*_, Label} to WikiFA where *Q*_*F*_ is the translation of *Q*_*E*_ in Persian, and *A*_*F*_ is the translation of *A*_*E*_ in Persian.  Figure 1 shows the production process of the WikiFA dataset.

### 3.2. PASD

There are some machine reading comprehension datasets for Persian [66, 67]. We build PASD by using the PersianQuAD dataset [67]. PersianQuAD is the first large-scale native machine reading comprehension dataset for question answering for the Persian language. It contains about 20000 questions posed by native annotators on a set of Persian Wikipedia articles. To build PersianQuAD, the annotators were shown the paragraphs of the Persian Wikipedia articles; then, they were asked to pose some questions on the paragraph and highlight the answer within the paragraph text. In order to use a question answering dataset to create an answer selection dataset, two challenges should be addressed:

1. In the question answering dataset, the answer to each question is within the paragraph, while for the answer selection dataset, candidate answers must be proper sentences.
2. In the question answering dataset, only the exact answer is specified for each question, while the answer selection dataset also requires incorrect candidate answers.

To address the first challenge, we retrieve the sentence that contains the answer, as the answer sentence. *answer_start* value indicates the start-index character of the exact answer in the paragraph. To detect the answer sentence, the paragraph first is tokenized to its sentences. Then, by aggregating the length of sentences, the sentence containing the *answer_start* value is considered the answer sentence. Algorithm 2 describes this process.

To address the second challenge, that is, to specify an incorrect candidate answer for each question, one can use random sentences from the corresponding paragraph, as incorrect candidate answers. However, these lead to low-quality incorrect answers. To produce a high-quality answer selection dataset, incorrect answers should be similar to correct answers, semantically and grammatically.

In this article, we present a retrieval-based approach to produce appropriate incorrect answers for each question. We first downloaded the Persian Wikipedia documents (https://dumps.wikimedia.org/fawiki/20201220/fawiki-20201220-pagesarticles-multistream.xml.bz2), which are used for building the PersianQuAD dataset. We extracted individual paragraphs from the documents by the wikiextractor library (https://github.com/attardi/wikiextractor). We then used the information retrieval component to retrieve the most relevant paragraphs to each question in PersianQuAD dataset. As for the retriever, we used the whoosh library (https://whoosh.readthedocs.io/en/latest) and implemented a passage retrieval component. It receives the Persian Wikipedia paragraphs and a question in the PersianQuAD dataset as inputs, and returns the top 10 paragraphs related to the question.  Figure 2 shows the procedure of retrieving relevant paragraphs to each question in the PersianQuAD dataset, using the passage retrieval component.

To extract the answer of the question from the retrieved paragraphs, we used the answer extraction component. We fine-tuned the MBERT model [16] on the PersianQuAD dataset and prepared a model to find the exact answers (https://github.com/BigData-IsfahanUni/PersianQuAD). By passing the question and the returned paragraphs to the model, it finds the exact answer in the paragraphs. After finding the exact answers in the paragraphs, we asked two human annotators to determine whether the extracted answers can be considered incorrect answers to the questions. Finally, we select four incorrect answers for each question.  Figure 3 shows the procedure of extracting candidate answer sentences using an MBERT QA model. The distribution of interrogative words of the PASD dataset is similar to the PersianQuAD dataset.  Table 3 shows statistics of the PASD dataset based on distributions.

Finally, we asked human annotators to determine the expected answer type (EAT) for each question in the PASD dataset. We used the coarse-grained EAT classes, which are commonly used as EATs [20]: HUM, LOC, ENTY, and NUM. HUM class shows that the question is looking for a person or an organization as an exact answer. In this regard, LOC is looking for a location, ENTY is looking for a product or an object, and NUM is looking for a date or a time.

Overall, in comparison with PersianQuAD whose records include a question and an exact answer, the records of PASD contain a question, an exact answer, an answer sentence, an annotated answer sentence, and an EAT. Moreover, each question has a correct answer and four incorrect answers. The PASD is generated for using in answer selection systems, while the PersianQuAD is appropriate for MRC systems. We demonstrate the statistics of the PASD and WikiFA datasets in Tables 4 and 5, respectively.

## 4. The Proposed Method

In this section, we present the PerAnSel method for answer selection task for the Persian language. As mentioned earlier, an IR-based QA system consists of four main components: (1) question processing, (2) information retrieval, (3) answer extraction, and (4) answer selection. First, the system receives a question from the user. In the first step, we extract the EAT [20] from the question and pass it to the answer processing component. In the second step, a retriever is used to retrieve the most relevant paragraphs to the question. In the third step, an answer extraction method is utilized to extract the candidate answers to the question from the retrieved paragraphs. Finally, in the fourth step, the PerAnSel selects the best answer from candidate answers' pool.  Figure 4 shows the architecture of the QA system and the PerAnSel method. Algorithm 3 shows the process of our system. The details of each step are explained in the following sections.

### 4.1. Question Processing

This component extracts EAT from the question. EAT shows the type of the answers to the questions [35]. For example, the EATs for the questions *who is the best soccer player in history?* and *where is the highest mountain in the world?* are Person and Location, respectively.

We implement a method based on the BERT language model to detect the EAT of the question. In this method, the question is passed to the kernel as an input sentence. Then, the [CLS] token output vector is transferred to a fully connected network. The hidden layer is ℍ_*QC*_ ∈ *ℝ*^1024^, and the output layer is *𝕆*_*QC*_ ∈ *ℝ*^4^. The output layer shows the EAT of the question.  Figure 5 shows the architecture of this method.

### 4.2. Information Retrieval

As mentioned earlier, the QA systems find the answer to each question in the web pages. To this end, some methods are proposed such as ad-hoc IR methods [68] and neural IR methods [69]. Recently, neural IR methods have been mostly used in QA systems. These methods encode the question and each paragraph using neural networks and generate a dense vector representation for the question and the paragraph. Then, the similarity between these inputs is measured. Finally, the most relevant paragraphs are returned.

### 4.3. Answer Extraction

To find candidate answers to the question, a machine reading comprehension method is used. To this end, a BERT language model for QA can be used. This method encodes the question and relevant paragraphs using the BERT model. Then, the output vector of each token of the relevant paragraph is passed to a fully connected network, and a score is measured for each token. Finally, based on the scores, the start span token and end span token are specified. The sentence that contains these tokens is returned as the candidate answer.

### 4.4. Answer Selection

The answer selection component selects the best answer among a set of candidate answers to the question. In this article, we propose the PerAnSel method. PerAnSel is an answer selection method presented for the Persian language. The PerAnSel method is a Siamese-based method based on pairwise ranking [33] and consists of three main components: (1) preprocessing, (2) sentence representation, and (3) relevance measurement. The preprocessing component gives higher priority to the candidate answer sentences, which have the same EAT as the question. The sentence representation component generates a meaningful vector for the question and the answer candidates. The relevance measurement component measures the relevance between the question and the candidate answer in the proposed method. The sentence representation components consist of two main components: (1) SOVWO and (2) OWO . In the following sections, we describe these components.

#### 4.4.1. Preprocessing

In this component, we deploy Hooshvare NER (https://github.com/hooshvare/parsner) to determine the NEs (Named Entities) in the candidate answer sentences. For example, *Messi was the best player of LaLiga in 2015* includes three entity types: person, organization, and time. The annotated sentence is shown in the following equation:

(7) $$\begin{array}{c} \overset{\text{Person}}{\overset{︷}{\text{Messi}}}\text{ was the best player of }\overset{\text{Organization}}{\overset{︷}{\text{LaLiga}}}\text{ in }\overset{\text{Time}}{\overset{︷}{2015}}\text{.} \end{array}$$

The answer selection component uses the EAT of the question and gives higher priority to the candidate answer sentences, which have the same EAT at the question within their NEs. To this end, the NEs in the candidate answer sentence should be mapped to the corresponding class in EATs.  Table 6 shows the mapping between EATs with the corresponding NEs in Hooshvare NER. This component then replaces all tokens of candidate answer sentence whose type is EAT with the *SPECIAL*_*TOKEN*_ token. Algorithm 4 indicates the preprocessing step in the answer selection.

#### 4.4.2. Sentence Representation

We prepare a method called PERSEL (*PER*sian *SEL*ection) to generate a dense vector representation for the question and the answer candidate. As shown in Figure 6, the PERSEL consists of SOVWO and OWO methods. In this method, we generate *𝕆*_SOVWO_ ∈ *ℝ*^600^ vector by using the SOVWO method and *𝕆*_OWO_ ∈ *ℝ*^600^ vector by using the OWO method. Then, *𝕆*_SentRep_ ∈ *ℝ*^600^ is generated based on Equation (8). *α* and *β* show the coefficient of SOVWO and OWO methods, respectively, for the Persian language. These coefficients are learned during training phase. Algorithm 5 shows the process of the sentence representation component.

(8) $$\begin{array}{c} O_{\text{SentRep}}=\alpha O_{\text{SOVWO}}+\beta O_{\text{OWO}}. \end{array}$$

*(1) SOVWO.* We examine SOVWO to show the performance of sequential models on sentences with SOV word order. This method is appropriate for standard word order such as SOV, because most sentences of the Persian language are stated in this order. As shown in Figure 7, the SOVWO method consists of a 1-D CNN and LSTM subcomponents. For the CNN subcomponent, the window size is 4, the padding value is 3, the number of filters is 300, and the pool function is also Max-pooling. Moreover, for the LSTM subcomponent, the hidden layer is ℍ_LSTM_ ∈ *ℝ*^300^ vector.

In the SOVWO method, the input sentence first is tokenized. We then present each token by its corresponding word embedding vector from pretrained fastText 300-dimensional vectors [70]. Afterward, we concatenate the word embedding vector of the input sentence's tokens and generate a matrix to represent the input sentence. Finally, this matrix is transferred as the input sentence representation to the CNN and the LSTM subcomponents. The output of the CNN subcomponent is *𝕆*_CNN_ ∈ *ℝ*^300^ vector, and the output of the LSTM subcomponent is *𝕆*_LSTM_ ∈ *ℝ*^300^ vector. By concatenating the output vectors of the subcomponents, *𝕆*_SOVWO_ ∈ *ℝ*^600^ vector is generated for the input sentence. Algorithm 6 shows the process of the SOVWO method.

*(2) OWO.* We examine OWO to deploy the power of fully connected neural networks and the attention mechanism for sentences with nonstandard word orders. This method is appropriate for all word orders such as SVO and OSV. As shown in Figure 8, this method utilizes an LSTM and a fully connected neural network. The hidden layer of the LSTM is a ℍ_LSTM_ ∈ *ℝ*^300^ vector.

In the OWO method, the kernel is the BERT language model. The input sentence is tokenized using Wordpiece or SentencePiece (We use Wordpiece for MBERT, DistilmBERT, ParsBERT; SentencePiece for AlbertFA). By passing these tokens to the BERT language model, *𝕋*_BERT_ ∈ *ℝ*^768^ is generated for each token. By concatenating these vectors, *𝕆*_BERT_ ∈ *ℝ*^|*S*|*∗*768^ is produced, each row of which is the output vector of an input token (|S| is length of the input sentence.). Afterward, we pass *𝕆*_BERT_ to the LSTM and take the *𝕆*_LSTM_ ∈ *ℝ*^300^. The *[CLS]* token output vector is passed to a fully connected neural network. The hidden layer is ℍ_[CLS]_ ∈ *ℝ*^1024^, and the output layer is *𝕆*_[CLS]_ ∈ *ℝ*^300^. Finally, we concatenate the output of *𝕆*_[CLS]_ vector and *𝕆*_LSTM_ and generate *𝕆*_OWO_ ∈ *ℝ*^600^ vector. Algorithm 7 shows the process of the OWO method.

#### 4.4.3. Relevance Measurement

This component measures the relevance between the question and the candidate answers. This method is composed of a fully connected neural network. In this component, we generate a value that specifies the relevance. To perform this, we concatenate the output of the sentence representation for the question and the candidate answer. Then, we pass this vector to a fully connected neural network. The hidden layer is ℍ_relevance_ ∈ *ℝ*^2048^, and the output layer is *𝕆*_relevance_ ∈ *ℝ*^1^. Algorithm 8 shows the process of the relevance measurement component.

## 5. Experiments

### 5.1. Baseline Models

As mentioned in Section 4, we proposed a method called PerAnSel for answer selection task for the Persian language. We consider four kernels for OWO method containing ParsBERT [64] and AlbertFA [65] for Persian, and DistilmBERT [48] and MBERT [16] as multilingual kernels. We compare this method to two baseline methods: (1) ASBERT and (2) CETE.

In the ASBERT [49], they focus on the ranking methods. They employ Siamese and triplet networks to encode input sentences by the BERT language model for answer selection tasks. In the CETE [45], they focus on the language models. They utilize language models such as ELMo, BERT, and RobertA to encode sentences for answer selection tasks.

### 5.2. Implementation Details

In order to implement the PerAnSel method, we used the PyTorch framework in Python 3.7. We trained and inferred the model in Google Colab (https://colab.research.google.com) environment on the NVIDIA Tesla T4 16 GB. The batch size is 8 and 4 for the question classifier and the answer selection method, respectively. The activation function is Gelu for language models and Relu for fully connected networks, LSTMs, and CNNs.

To train models, we consider the learning rate 1*e*^−2^ and train the proposed model on 4 epochs for the question classifier and 2 for the answer selection method. WarmupLinearSchedular [71] is used to schedule the learning rate. WarmupLinearSchedular is a learning rate schedule where the learning rate increases linearly from a low rate to a constant rate thereafter. This reduces volatility in the early stages of training. The AdamW optimizer is used to train all models.  Table 7 shows the number of training parameters of the methods. The training time of the models is shown in Table 8.

In order to evaluate the question classifier, we used the accuracy metric. Accuracy shows the proportion of correct predictions to the whole number of predictions. Equation (9) shows the accuracy metric. To evaluate the answer selection method, we used the MRR metric. The MRR is a measure for evaluating methods, which generates a list of possible responses to some queries, ordered by relevancy [21]. The reciprocal rank of a query response is the multiplicative inverse of the rank of the first relevant answer: 1 for first place, 1/2 for second place, 1/3 for third place, and so on. The mean reciprocal rank is the average of the reciprocal ranks of results for queries. In our system, the queries are the questions, and the responses are the relevant answers. Equation (10) shows this metric:

(9) $$\begin{array}{c} \text{Acc}\left(Q\right)=\frac{\text{Number of correct predictions }\left(Q\right)}{\text{Total of all cases to be predicted}\left(Q\right)}, \end{array}$$

(10) $$\begin{array}{c} \text{MRR}\left(Q\right)=\frac{1}{\left|Q\right|}\sum_{j=1}^{\left|Q\right|}r_{j}. \end{array}$$

In Equations (9) and (10), *Q* shows the questions in the dataset. *r*_*j*_ is also the inverse of the first rank of the *q*_*j*_ answer.

## 6. Results and Discussion

### 6.1. Answer Selection

In this article, we present PASD, the first large-scale native answer selection dataset. We also present the PerAnSel method to solve the answer selection problem for the Persian language: (1) SOVWO, (2) OWO, and (3) PERSEL. For methods that use BERT inside them (OWO and PERSEL), we examined four versions of the BERT (ParsBERT, AlbertFA, DistilmBERT, and MBERT) in each model. Hence, we build eight BERT-based answer selection systems according to the core answer selection method and BERT-version examined.  Table 9 shows the description of the systems.

We also implement two baseline systems: (1) ASBERT and (2) CETE. We train each of the answer selection systems using the training set of the datasets and evaluate them with the test set. We evaluate each of the answer selection systems according to MRR measurement described in Section 5.2.  Table 10 and Figure 9 show the performance of the answer selection systems on WikiFA, PerAnSel, and PerCQA [60] datasets, respectively. We also show the *α* and *β* for the PERSEL method in Table 11.

We derive the following observations from the results:

- *The SVOWO method has the worst performance than the other proposed methods.*
- This is because of the lack of model knowledge from the language and the answer selection task. The method consists of CNN and LSTM networks with no prior knowledge and has training parameters with random weights.
- *The OWO and PERSEL methods performance is improved by transferring the kernel to ParsBERT, AlbertFA, DistilmBERT, and MBERT, respectively.*
- This is because of the quality and the volume of the information, which is used to train the language models.
- *The PERSEL method has the best performance.*
- We hypothesize that this method supports all kinds of word orders such as SOV, SVO, and OSV. The SOVWO processes SOV word order and the BERT component processes other word orders.
- *The OWO and PERSEL method have better performance than the CETE method.*
- This is because using the *[CLS]* token output of the BERT language model has more unsatisfactory performance than using the output vector of all token outputs.
- *The OWO-MBERT and PERSEL-MBERT have better performance than the ASBERT method.*
- We hypothesize that this can be attributed to the fact that using pairwise ranking and Siamese architecture performs better than the mere use of Siamese architecture merely.
- *Experimental results on WikiFA and PASD datasets show that the performance of the native dataset (PASD) is better than the translated dataset (WikiFA).*
- This is because the quality of the dataset language significantly impacts the accuracy and performance of the answer selection system.
- *Despite the fact that PASD and PerCQA are native datasets, the experimental results show that models have better performance on PASD than PerCQA.*
- We hypothesize that this can be attributed to the fact that deep learning models require amount of annotated data for training to have acceptable performance.
- *Experimental results on the WikiFA dataset show that unlike PASD and PerCQA, α is less than β*.
- We hypothesize that this is because that the words of translated sentences are in various orders than native sentences, which mostly are in the SOV word order.
- *The α and β are closer together for t*he *PerCQA dataset than the PASD dataset.*
- This is because the language of PerCQA is informal Persian and the language of PASD is formal Persian. In the PASD dataset, native annotators try to compose sentences in standard word order (SOV). So, the effect of SOVWO is more significant than OWO.

### 6.2. Question Classifier

In Section 3, we presented the PASD dataset to be used in answer selection task. In Section 3.2, we enhanced the dataset for question processing and also presented a question classifier, which use PASD as the training set and classifies the questions. In this section, we evaluate the question classifier both intrinsically and extrinsically. In intrinsic evaluation, we measure the performance of the question classifier in terms of accuracy. In extrinsic evaluation, we measure the impact of the question classifier on the answer selection task.  Table 12 shows the accuracy of the question classifier with four kernels examined and trained on the PASD dataset.

Table 12 shows that by using MBERT as the kernel of the question classifier, the best accuracy is obtained. This can be attributed to the quality and the volume of the information that is used to train the language models.  Table 12 indicates that monolingual language models such as ParsBERT and AlbertFA have less accuracy than multilingual language models such as DistilmBERT and MBERT. Moreover, the superiority of MBERT rather than DistilmBERT can be attributed to the number of learnable parameters.

In order to measure the impact of the question classifier component on answer selection task, as mentioned in Section 4.4.1, we utilize the output of the question processing in answer selection systems.  Table 13 shows the performance of the answer selection systems, using the question classifier component on PASD, PerCQA, and WikiFA datasets. As for question classifier kernel, we used MBERT, which shows the best performance.

Here we observe:

- *The performance of BERT-based methods is better than non-BERT methods.*
- *Combining the question classifier with the PERSEL method performs best.*
- *The performance of the model on the WikiFA dataset is reduced by combining the question processing component*

 We hypothesize that this can be attributed to the fact that the detection of the EAT for automatically translated sentences in WikiFA is more challenging than native sentences, because the syntactic and semantic structures of translated sentences are low quality.

### 6.3. Error Analysis

In this section, we analyze errors of the question classifier and answer selection method and indicate which interrogative words these methods are compatible with.  Table 14 shows the error analysis on question classifier, and Table 15 shows the error analysis results on the PERSEL method on the PASD dataset.

According to Tables 14 and 15, and Figure 10, we observe the following:

- Table 14* shows the most error is related to the why word.*
-  Because there is no corresponding EAT to *why* questions. In other words, the exact answer of *why* questions is a multiword expression, which is not equal to any EATs. Also, answering this type of question requires reason and logic.
- Table 15* shows that using the question processing component is very effective in answering some questions.*
- Because the MRR of six interrogative words (what, how, when, where, who, which) is improved rather than a system without using the question classifier.
- Figure 10* demonstrates that the MRR measure for each interrogative word is improved, except for whyword.*

 This is because the exact answer of*why* questions is a multiword expression, which is not equal to any EATs.

## 7. Conclusion

In this article, we present the first large-scale native answer selection dataset for the Persian language called PASD. We also propose an answer selection model called PerAnSel for the answer selection task in Persian QA systems. Evaluating PerAnSel on the Persian language shows the superiority of PerAnSel over the state-of-the-art methods. The Persian language is a free word-order language. The standards word order in Persian is SOV, but other word orders are also correct. In PerAnSel, we parallelize a sequential and a transformer-based method to handle various orders in the Persian language. The results show that sequential models such as LSTM and 1-D CNN work better on standard word order (SOV) and transformer-based models such as BERT language models composed of fully connected networks and attention mechanism works well for other word-order types, in the Persian language. As for future work, we can mention the use of generative methods to generate datasets [72]. In these methods, in addition to the translation and native datasets, an automated dataset produced by generative methods can be employed.

## Figures and Tables

**Figure 1:** For each record, *R*_*E*_={*Q*_ID, *Q*_*E*_, *D*_ID, *D*_Title, *A*_ID, *A*_*E*_, Label}, where *Q*_ID is question id, *Q*_*E*_ is a question in English, *D*_ID is the document id, *D*_Title is the document title, *A*_ID is the candidate answer id, *A*_*E*_ is a candidate answer in English, and Label is the candidate answers' label, and a record *R*_*F*_={*Q*_ID, *Q*_*F*_, *D*_ID, *D*_Title, *A*_ID, *A*_*F*_, Label} is added to WikiFA, where *Q*_*F*_ and *A*_*F*_ are the translations of *Q*_*E*_ and *A*_*E*_ in Persian (orange arrows), respectively.

**Figure 2:** (1) Paragraphs are indexed by the Whoosh library, (2) The ten most relevant paragraphs are retrieved for each question of the PersianQuAD dataset.

**Figure 3:** (1) An MBERT language model is fine-tuned on PersianQuAD. (2) Each question of PersianQuAD dataset and its relevant paragraphs are passed to the fine-tuned MBERT. (3) The correct sentence answer and its corresponding paragraph are added to the PASD as correct candidate answer (orange arrow). (4) The four most relevant incorrect answer and their corresponding paragraph are also added as incorrect candidate answers.

**Figure 4:** In this figure, green components indicate the main components of PerAnSel model. Orange, red, and dark-green vectors show the output of [CLS] token, CNN, and RNN networks respectively. (1) The question is passed to the Question Processing and the EAT is detected. (2) In the information retrieval, the most relevant paragraphs to the question are retrieved from documents. (3) The question and its relevant paragraphs are transferred to the Answer Extraction to find the exact answer from each paragraph. (4) The EAT, the question, and extracted exact answers are passed to the Answer Selection, and (5) the most correct answer is returned to the user (violet).

**Figure 5:** (1) The question is passed to a pretrained MBERT. (2) The [CLS] token (orange) is sent to a fully connected network. (3) The EAT is detected as the output.

**Figure 6:** (1) The input sentence is passed to the SOVWO and OWO components. (2) The output vectors of the SOVWO (red and green) and OWO (blue and green) components are summed. (3) The final vector is returned as output.

**Figure 7:** (1) The input sentence is passed to a CNN and RNN component. (2) The output vectors (red for CNN and green for RNN) are concatenated. (3) The final vector is returned as output.

**Figure 8:** (1) The sentence is passed to a pretrained MBERT. (2) The [CLS] token (orange) is sent to a fully connected network. (3) Other tokens are sent to a LSTM network (green). (4) The output of LSTM and fully connected network are concatenated. (5) The final vector is returned as output.

**Figure 9:** The MRR measure of the PerAnSel method on PASD, PerCQA, and WikiFA datasets.

**Figure 10:** The MRR results of interrogative words.

**Algorithm 1:** Algorithm of BERT language model.

**Algorithm 2:** Extracting answer sentence from candidate paragraphs.

**Algorithm 3:** The process of the IR-based QA system.

**Algorithm 4:** Preprocessing step of the answer selection.

**Algorithm 5:** The processing of the PERSEL.

**Algorithm 6:** The process of the SOVWO method.

**Algorithm 7:** The process of the OWO method.

**Algorithm 8:** The processing of the relevance measurement.

**Table 1:** Review of answer selection datasets for various languages.

Dataset	Language	Type	Domain	Train	Dev	Test
TrecQA (raw) [23]	English	Native	Open	1229/94	82	100
TrecQA (clean) [24]	English	Native	Open	1229/94	65	68
WikiQA [18]	English	Native	Open	2118	396	633
InsuranceQA [25]	English	Native	Close	12889	2000	2000
SelQA [26]	English	Native	Open	5529	785	1590
cMedQA v1 [53]	Chinese	Native	Close	50000	2000	2000
cMedQA v2 [54]	Chinese	Native	Close	100000	4000	4000
cEpilepsyQA [55]	Chinese	Native	Close	3920	490	490
DBQA [56]	Chinese	Native	Open	8772	4779	2500
MilkQA [57]	Portuguese	Native	Close	2307	50	300
WikiQAar [58]	Arabic	Translation	Open	2118	396	633
CQA-MD [59]	Arabic	Native	Close	1031	250	250
PerCQA [60]	Persian	Native	Open	692	99	198
PASD	Persian	Native	Open	**17567**	**1000**	**1000**

The bold row indicates our new dataset.

**Table 2:** A summary of answer selection models for various languages. In this table, PP refers to preprocessing, LR refers to low resource, MR refers to morphologically rich, FWO refers to free word order, and RTL refers to right to left.

No.	Paper	Year	Architecture	Language	Network	PP	LR	MR	FWO	RTL
1	Wan et al. [27]	2006	Feature Engineering	English	Tree	✓	*χ*	*χ*	*χ*	*χ*
2	Punyakanok et al. [29]	2004	Feature Engineering	English	Tree	✓	*χ*	*χ*	*χ*	*χ*
3	Heliman and Smith [30]	2010	Feature Engineering	English	Tree	*χ*	*χ*	*χ*	*χ*	*χ*
4	Yu et al. [32]	2014	Siamese	English	CNN	*χ*	*χ*	*χ*	*χ*	*χ*
5	He et al. [33]	2015	Siamese	English	CNN	*χ*	*χ*	*χ*	*χ*	*χ*
6	Rao et al. [34]	2016	Siamese	English	CNN	*χ*	*χ*	*χ*	*χ*	*χ*
7	Kamath et al. [35]	2019	Siamese	English	RNN	✓	*χ*	*χ*	*χ*	*χ*
8	Yang et al. [36]	2016	Attention	English	CNN	*χ*	*χ*	*χ*	*χ*	*χ*
9	He et al. [37]	2016	Attention	English	CNN	*χ*	*χ*	*χ*	*χ*	*χ*
10	Mozafari et al. [38]	2019	Attention	English	CNN	✓	*χ*	*χ*	*χ*	*χ*
11	He and Lin [40]	2016	Compare-Aggregate	English	CNN, RNN	*χ*	*χ*	*χ*	*χ*	*χ*
12	Wang et al. [41]	2017	Compare-Aggregate	English	RNN	*χ*	*χ*	*χ*	*χ*	*χ*
13	Yoon et al. [42]	2019	Language Model	English	Elmo	*χ*	*χ*	*χ*	*χ*	*χ*
14	Mozafari et al. [44]	2019	Language Model	English	Bert, RNN	✓	*χ*	*χ*	*χ*	*χ*
15	Laskar et al. [45]	2020	Language Model	English	Bert, RobertA	*χ*	*χ*	*χ*	*χ*	*χ*
16	Mozafari et al. [47]	2020	Language Model	English	DistilBERT	✓	*χ*	*χ*	*χ*	*χ*
17	Shonibare [49]	2021	Language Model	English	Bert, RobertA	*χ*	*χ*	*χ*	*χ*	*χ*
18	Han et al. [50]	2021	Language Model	English	RobertA	*χ*	*χ*	*χ*	*χ*	*χ*
19	Shen et al. [51]	2018	Other	English	CNN, RNN	✓	*χ*	*χ*	*χ*	*χ*
20	Jin et al. [52]	2020	Others	English	CNN, RNN	*χ*	*χ*	*χ*	*χ*	*χ*
21	Zhang et al. [54]	2018	Attention	Chinese	CNN, RNN	✓	✓	✓	✓	*χ*
22	Zhang et al. [61]	2019	Siamese	Chinese	CNN, RNN	✓	✓	✓	✓	*χ*
23	Chen et al. [55]	2021	Attention	Chinese	CNN	✓	✓	✓	✓	*χ*
24	Almiman et al. [62]	2020	Language Model	Arabic	Bert	✓	✓	✓	*χ*	✓
25	PerAnSel	2022	Language Model	Persian	Bert, CNN, RNN	✓	✓	✓	✓	✓

**Table 3:** The statistics of the PASD dataset. The first row shows the number of questions in train set and test set.

Interrogative word	Train/Dev	Test
	18567	1000
What	28.57%	23.2%
How	15.54%	13.2%
When	11.0%	8.30%
Where	13.21%	21.1%
Who	16.13%	13.0%
Which	14.61%	20.7%
Why	0.94%	0.60%

**Table 4:** The statistics of the PASD datasets.

	Train	Dev	Test
# of questions	17567	1000	1000
# of sentences	87835	5000	5000
Avg. len. of ques.	10.77	10.41	10.46
Avg. len. of sent.	21.66	32.63	32.08

**Table 5:** The statistics of the WikiFA datasets.

	Train	Dev	Test
# of questions	2117	296	630
# of sentences	20347	2733	6116
Avg. len. of ques.	7.14	7.16	7.17
Avg. len. of sent.	27.21	26.16	26.67

**Table 6:** Fine-grained and coarse-grained entity types.

EAT	Equivalent NE in NER
HUM	PERSON, ORGANIZATION
LOC	LOCATION
ENTY	PRODUCT, EVENT, FACILITY
NUM	DATE, TIME, PERCENT, MONEY

**Table 7:** Number of training parameters of Question Classifier, SOVWO, OWO, and PERSEL methods as sentence representation. The notation k indicates Kilo.

LM					
Method	—	ParsBERT	AlbertFA	DistilmBert	MBERT
SOVWO	8100 k	—	—	—	—
Question classifier	—	110000 k	110000 k	66000 k	179000 k
OWO	—	115956 k	16956 k	71956 k	184956 k
PERSEL	—	119036 k	20036 k	75036 k	188036 k

**Table 8:** Training time of the question classifier and sentence representation methods. The notation m shows minute.

LM					
Method	—	ParsBERT	AlbertFA	DistilmBert	MBERT
SOVWO	6 m	—	—	—	—
Question classifier	—	140 m	15 m	75 m	270 m
OWO	—	160 m	25 m	90 m	310 m
PERSEL	—	170 m	30 m	95 m	320 m

**Table 9:** The implemented QA system with their descriptions.

System	Description
ASBERT	Shonibare [49]
CETE	Rahman Laskar et al. [45]
SOVWO	A method using LSTMs and CNNs
OWO-ParsBERT	OWO method with ParsBERT kernel for Persian
OWO-AlbertFA	OWO method with AlbertFA kernel for Persian
OWO-DistilmBERT	OWO method with DistilmBERT kernel
OWO-MBERT	OWO method with MBERT kernel
PERSEL-ParsBERT	PERSEL method with ParsBERT kernel in the LM component for Persian
PERSEL-AlbertFA	PERSEL method with AlbertFA kernel in the LM component for Persian
PERSEL-DistilmBERT	PERSEL method with DistilmBERT kernel in LM component
PERSEL-MBERT	PERSEL method with MBERT kernel for BERT component

**Table 10:** The MRR measure of the PerAnSel method on PASD, PerCQA, and WikiFA.

System	Dataset		
	PASD (%)	PerCQA (%)	WikiFA (%)
ASBERT-MBERT	81.45	64.69	51.32
CETE-MBERT	79.99	61.36	42.74
SOVWO	70.48	52.28	30.84
OWO-ParsBERT	72.15	55.68	43.46
OWO-AlbertFA	75.36	58.21	48.47
OWO-DistilmBERT	77.98	61.02	50.36
OWO-MBERT	82.14	66.47	52.96
PERSEL-ParsBERT	74.30	55.97	50.38
PERSEL-AlbertFA	77.21	59.78	47.59
PERSEL-DistilmBERT	81.55	65.44	62.66
PERSEL-MBERT	89.36	69.48	66.08

**Table 11:** The *α* and *β* of the PERSEL method.

Dataset factor	Factor	
	*α*	*β*
PASD	0.74	0.26
PerCQA	0.61	0.39
WikiFA	0.35	0.65

**Table 12:** The accuracy of question classifiers.

Model	PASD (%)
ParsBERT	88.2
AlbertFA	90.7
DistilmBERT	95.3
MBERT	97.9

**Table 13:** The MRR of combining the question classifier with the answer selection component on MBERT.

Method	PASD (%)	PerCQA (%)	WikiFA (%)
SOVWO	71.22	56.27	25.71
OWO	85.99	70.12	50.74
PERSEL	92.11	73.11	62.77

**Table 14:** Error analysis on the question processing component.

Interrogative word	Percent	Accuracy (%)
What	23.2	97.8
How	13.2	95.4
When	8.30	98.7
Where	21.1	99.5
Who	13.0	98.4
Which	20.7	99.5
Why	0.60	16.6

**Table 15:** Error analysis on the PERSEL method.

Interrogative word	Percent	MRR without QC (%)	MRR with QC (%)
What	23.2	84.9	91.8
How	13.2	85.6	93.9
When	8.30	90.3	96.3
Where	21.1	93.3	98.1
Who	13.0	91.5	97.6
Which	20.7	94.6	99.0
Why	0.60	16.6	16.6

## Data Availability

Data used to support the findings of this study are available from the GitHub Repository at https://github.com/BigData-IsfahanUni/PerAnSel and https://github.com/PerCQA/PerCQA-Dataset.
